The article "Impact of Intraspinal Nerve Block Anesthesia on Intrapartum Fever and the Neonate" was retracted in 2023. Reasons: suspected computer-generated content; unreliable results or conclusions; concerns about the data; concerns about the results or conclusions.

# Impact of Intraspinal Nerve Block Anesthesia on Intrapartum Fever and the Neonate

**DOI:** 10.1155/2022/2600755

**Published:** 2022-05-29

**Authors:** Lei Wang, Ruijie Chang, Xinyan Chen

**Affiliations:** ^1^Department of Surgical Anesthesia, Shiyan Maternal and Child Health Care Hospital, Hubei Medical College, Shiyan, China; ^2^Department of Anesthesiology, Taihe Hospital, Hubei Province, Shiyan, China

## Abstract

**Objective:**

To evaluate the impact of intraspinal nerve block anesthesia on intrapartum fever and the neonate.

**Methods:**

In this prospective study, between October 2019 and December 2020, 90 eligible primiparous women enrolled in the obstetrics and gynecology department of our hospital for delivery were recruited and assigned via the random number table method at a ratio of 1 : 1 to either an analgesic group given intraspinal nerve block anesthesia for labor or a nonanalgesic group without anesthesia for labor. Outcome measures included intrapartum body temperature, cases of intrapartum fever, Apgar scores of neonates, visual analogue scale (VAS) scores, delivery mode, and indomethacin use.

**Results:**

Intraspinal nerve block anesthesia was associated with a higher body temperature at 4 h and 5 h after analgesia and more cases of intrapartum fever versus no anesthesia (*P* < 0.05). There were no significant differences in the Apgar scores between the two groups (*P* > 0.05). Participants given intraspinal nerve block anesthesia had lower VAS scores during labor versus those without anesthesia (*P* < 0.05). The differences in the delivery mode between the two groups were not significant (*P* > 0.05). Intraspinal nerve block anesthesia resulted in a significantly higher demand for indomethacin versus no anesthesia (*P* < 0.05).

**Conclusion:**

Intraspinal nerve block anesthesia is clinically effective in labor analgesia but may cause increased body temperature or even overt clinical fever, so close clinical observation of maternal temperature changes is required to mitigate the effects of anesthesia on the mothers. No adverse consequences of intraspinal nerve block anesthesia on the newborns were reported in this study.

## 1. Introduction

The severe pain of vaginal delivery [1] may cause negative emotions such as fear and worry, and may also result in syncope, weakness, and even fetal distress, cesarean section, and fetal death in severe cases [2]. Labor pain will elicit physiological stresses and perinatal complications [3]. Pregnant women choose cesarean delivery due to the fear of labor pain, which is one of the important influencing factors for the increasing rate of cesarean delivery in China [4]. Intraspinal nerve block anesthesia for labor analgesia features satisfactory nerve block and ideal analgesic effect, but the uncertainty of its effect on the labor process and the fetus has prevented its widespread implementation in China [5]. Epidural analgesia is associated with a significantly elevated incidence of intrapartum fever [2]. Intradural labor analgesia causes antepartum noninfectious fever, probably because epidural anesthesia dilates the limb vessels below the plane of anesthesia to increase convective radiation heat dissipation, and reduces skeletal muscle activity to decrease thermogenesis. In addition, the asynchrony of anesthesia on cold and heat sensory blocks leads to early onset of thermothermal block and deviation of body temperature information from the thermoregulatory center, resulting in elevated body temperature during labor [2]. However, fever due to intralesional analgesia does not usually exceed 38°C, and fever above 38°C is associated with chorioamnionitis. Accordingly, 90 eligible primiparous women enrolled in the obstetrics and gynecology department of our hospital for delivery were recruited to evaluate the impact of intraspinal nerve block anesthesia on intrapartum fever and the neonate and to provide a reference for further treatment. Traditional Chinese medicine (TCM) acupressure is a traditional Chinese medical practice that can be used to relieve patients' negative emotions and reduce pain by stimulating different acupuncture points.

## 2. Materials and Methods

### 2.1. Baseline Profile

In this prospective study, between October 2019 and December 2020, 90 eligible primiparous women in the obstetrics and gynecology department of our hospital for delivery were recruited and assigned via the random number table method at a ratio of 1 : 1 to either an analgesic group given intraspinal nerve block anesthesia for labor or a nonanalgesic group without anesthesia for labor. The clinical features of the analgesic group (aged 20–32 years, a mean age of 25.61 ± 2.72 years, a height of 153–172 cm, a mean height of 162.27 ± 5.46 cm, a weight of 51–77 kg, mean weight of 60.17 ± 7.76 kg, gestational week of 38–41 weeks, mean gestational week of 39.26 ± 1.72 weeks) were comparable with those of the nonanalgesic group (aged 20–33 years, mean age of 25.70 ± 2.68 years, a height of 151–173 cm, a mean height of 162.54 ± 5.31 cm, a weight of 50–75 kg, mean weight of 60.31 ± 7.68 kg, gestational week of 38–41 weeks, mean gestational week of 39.33 ± 1.70 weeks) (*P* > 0.05) (Table 1). The study was certified by the Ethics Committee of Shiyan Maternal and Child Health Care Hospital, with ethics certificate number 2018-11-15. All mothers and families signed the informed consent form.

### 2.2. Inclusion and Exclusion Criteria

Inclusion criteria are as follows: subjects who met the criteria of American Society of Anesthesiologists (ASA) class I-II; with no contraindications to intralesional anesthesia; with a singleton; with a full-term pregnancy; and with a primary birth were included.

Exclusion criteria are as follows: subjects with comorbid metabolic diseases, such as diabetes mellitus; with a basal body temperature higher than 37.5°C; and with high-risk pregnancies were excluded.

### 2.3. Treatment Method

Subjects in the nonanalgesic group underwent normal labor. In the analgesic group, the subjects were anesthetized by intraspinal nerve block. After the determination of labor, the epidural puncture was performed at L2∼3. After the puncture needle entered the epidural cavity, a 4 cm epidural catheter was placed cephalad to the side of the head and secured. After the injection of 3 mL of 2% lidocaine and observation for 5 min to confirm the absence of maternal subarachnoid block and symptoms of local anesthetic toxicity, 3–5 mL of 1.5% lidocaine was given with the plane of anesthesia controlled below T10. Subjects in the analgesic group received an electronic analgesia pump to administer a mixture of 0.1% ropivacaine + 0.5 *μ*g/mL fentanyl, at a background dose of 5–10 mL/h depending on maternal weight, and self-administered analgesia (PCA) dose of 2–5 mL/dose with a lockout time of 15 min. The ideal dose was to achieve the best pain control during contractions and to preserve the subjects' feeling of slight uterine contractions. The maternal analgesic planes and pain degree were tested, the maternal motor nerve block was graded, and the maternal vital signs were monitored, with continuous fetal heart monitoring. The women were encouraged to rest and mobilize from bed, which facilitated the progress of labor and the descent of the fetal previa. After delivery, the women were monitored in the delivery room for 2 h, and the epidural catheter was removed on departure from the delivery room.

Patients in both groups were given TCM acupressure. The TCM rehabilitation physiotherapy center trained the physiotherapists in acupressure, including acupoint identification, massage techniques, and acupressure duration. Pain in the small abdomen is mostly seen in the first stage of labor, while pain in the lower back is mostly seen in the second stage of labor. For small abdominal pain, Guanyuan point, Qihai point, and Zhongji point were used as the main points for acupressure, and the above points with the Hegu, Sanyin, and Kunlun points were jointly massaged. For low back pain, the Ciliao point was used as the main acupoint, and the back and lumbosacral areas were massaged, followed by a massage of the hip with the Huantiao point as the main acupoint. For lumbosacral pain, a massage was performed along both sides of the spine with Shenyu, Guanyuanyu, E'shi, Neiguan, and Taichong points as the central points. In the massage, the massage points, strength, and techniques were timely adjusted according to the feedback of the subjects.

### 2.4. Outcome Measures

1. The maternal temperature and the number of fever cases after labor analgesia were recorded.
2. Neonatal Apgar score [6]: the neonatal Apgar score was used to assess neonatal asphyxia and hypoxia. The assessment includes five domains of skin color, heart rate, response to stimulation, muscle tone, and respiration, each with a score of 0–2 points and a total of 10 points. The assessment was performed at 1, 5, and 10 minutes postnatally. A score of 8–10 points is considered normal, a score of 4–7 points is mild asphyxia, and a score of 0–3 points is severe asphyxia. The 1-minute score reflects the severity of neonatal asphyxia and hypoxia, and the 5-minute score reflects the effect of resuscitation after neonatal asphyxia and hypoxia, which facilitates the judgment of the prognosis.
3. Visual analogue scale (VAS) score [7]: the VAS score was used to assess the pain, with 0 points for no pain, 1–3 points for mild pain, 4–6 points for moderate pain, and 7–10 points for severe pain. The higher the scores, the more severe the pain.
4. The mode of delivery and the use of indomethacin was recorded.

### 2.5. Statistical Analysis

SPSS 22.0 was used for data analyses, and GraphPad Prism 8 was used to plot the data. The measurement data are expressed as (mean ± SD) and analyzed using the independent sample *t*-test. The count data are expressed as the number of cases (rate) and analyzed using the chi-square test. Differences were considered statistically significant at *P* < 0.05.

## 3. Results

### 3.1. Body Temperature and Cases of Intrapartum Fever

Intraspinal nerve block anesthesia was associated with a higher body temperature at 4 h and 5 h after analgesia and more cases of intrapartum fever versus no anesthesia (*P* < 0.05) (Table 2).

### 3.2. Apgar Score

There were no significant differences in the Apgar scores between the two groups (*P* > 0.05) (Figure 1).

### 3.3. VAS Score

Subjects given intraspinal nerve block anesthesia showed lower VAS scores throughout the labor process versus those without anesthesia (*P* < 0.05) (Table 3).

### 3.4. Delivery Mode and Indomethacin Use

The differences in the delivery mode between the two groups were not significant (*P* > 0.05). Intraspinal nerve block anesthesia resulted in a significantly higher demand for indomethacin versus no anesthesia (*P* < 0.05) (Table 4).

## 4. Discussion

The process of labor includes uterine contractions, receding of the canal, dilatation of the uterine opening, the descent of the fetal previa, and delivery of the fetus [6], during which the pulling of the cervix and the dilation of the delivery canal may cause severe pain [7]. In addition, the intense tension, fear, and anxiety of pregnant women during labor may aggravate the women's sensitivity to pain. Severe pain seriously interferes with normal delivery and may threaten the life of the fetus in severe cases [8]. Thus, the exploration for safe and painless labor remains one of the key clinical issues to be addressed. Currently, clinical research has concluded that intraspinal nerve block anesthesia is the safest and most effective method of analgesia for labor [9]. It reduces maternal pain by blocking the sensory nerves that innervate the uterus in the body through intermittent or continuous infusion of local anesthetic drugs and analgesic drugs into the spinal canal. Due to the small amount of anesthesia used, the women can still feel the contractions [10]. Qiu et al. revealed that the analgesic effect of epidural self-administered analgesic pump analgesia is favorable with rapid efficacy [11], and the placenta is less affected by the drug, which indicates the safety of the fetus during delivery [12]. However, clinical studies have revealed a significant increase in body temperature or even overt clinical fever in women given intraspinal nerve block anesthesia. A large body of evidence supports that intrapartum fever after intraspinal nerve block anesthesia is a noninfectious inflammation [13]. He et al. [14] noted that the emergence of maternal fever after the administration of intraspinal nerve block anesthesia was mainly seen at 3–5 h after analgesia, where the dose of anesthetic drugs contributes most to the maternal temperature changes. In addition, the prolongation of the maternal survival process is also considered an independent influencing factor of intrapartum fever. Therefore, the avoidance of prolonged labor is considered an effective measure for body temperature management [15].

In the present study, intraspinal nerve block anesthesia was associated with a higher body temperature at 4 h and 5 h after analgesia and more cases of intrapartum fever versus no anesthesia, indicating a negative impact of intraspinal nerve block anesthesia on maternal body temperature during labor [16]. The benefits of labor analgesia include no interference with the safety of the mother and fetus, no disruption of labor and contractions, simple administration, fast onset of action, and participation of the pregnant woman in the whole process of labor [17]. Epidural self-administered analgesia pump analgesia is considered a preferred method of labor analgesia [18]. However, it is associated with overt clinical fever during labor, which severely compromises the pregnant woman's body condition. Furthermore, maternal fever in labor decreases the sensitivity of the cervix and uterus to indomethacin, and weak contractions result in delayed cervical dilation, leading to a prolonged labor process or even obstructed labor [19]. Therefore, clinical attention to women with elevated body temperature and fever should be strengthened to minimize or avoid adverse maternal outcomes [20]. Here, the Apgar scores showed no significant differences between the two groups. However, the study by Liu et al. noted that high maternal body temperature may be associated with reduced pulmonary tone and neonatal asphyxia in the newborn [21]. In addition, no significant difference was found in the delivery mode, and intraspinal nerve block anesthesia resulted in a significantly higher demand for indomethacin versus no anesthesia, indicating the impact of intraspinal nerve block anesthesia analgesia on maternal contractions. Moreover, the subjects given intraspinal nerve block anesthesia showed lower VAS scores throughout the labor process versus those without anesthesia, suggesting a better analgesic effect of intraspinal nerve block anesthesia. The reason may be that the analgesic blocking plane is adjusted according to body position, thus allowing low concentrations of small doses of local anesthetic drugs to achieve the expected blocking plane with a fast onset of action and strong analgesic effect.

Acupressure is a common external therapeutic technique in TCM, by stimulating acupuncture points using massage techniques to produce therapeutic effects for corresponding body parts. Acupressure promotes the smooth flow of maternal meridians and local Qi and blood, regulates the function of internal organs and uterine status, reduces pain, and thus contributes to a smooth delivery [8].

## 5. Conclusion

Intraspinal nerve block anesthesia is clinically effective in labor analgesia but may cause increased body temperature or even overt clinical fever, so close clinical observation of maternal temperature changes is required to mitigate the effects of anesthesia on the mothers. No adverse consequences of intraspinal nerve block anesthesia on the newborns were reported in this study. The limitations of this study are the absence of long-term follow-up and the lack of investigation of the intellectual development of the children. The trial will be extended in the future with long-term follow-up to obtain more reliable data.

## Figures and Tables

**Figure 1:** Comparison of Apgar scores of the neonate. The comparison is not statistically significant (*P* > 0.05).

**Table 1:** Comparison of baseline profile.

	Analgesic group (*n* = 45)	Nonanalgesic group (*n* = 45)	*t*-value	*P* value
Age (year)	25.61 ± 2.72	25.70 ± 2.68	−0.158	0.875
Height (cm)	162.27 ± 5.46	162.54 ± 5.31	−0.238	0.812
Weight (kg)	60.17 ± 7.76	60.31 ± 7.68	−0.086	0.932
Gestational week (week)	39.26 ± 1.72	39.33 ± 1.70	−0.194	0.847

**Table 2:** Comparison of body temperature and cases of intrapartum fever.

Groups	*n*	1 h (°C)	2 h (°C)	3 h (°C)	4 h (°C)	5 h (°C)	Cases of intrapartum fever
Analgesic group	45	36.7 ± 0.4	36.7 ± 0.5	36.9 ± 0.5	37.6 ± 0.6	37.8 ± 0.5	9 (20%)
Nonanalgesic group	45	36.6 ± 0.5	36.6 ± 0.4	36.8 ± 0.4	36.8 ± 0.5	36.7 ± 0.5	0 (0%)
*t* or *x*^2^	—	1.048	1.048	1.048	6.871	10.436	10.000
*P* value	—	0.297	0.297	0.297	<0.01	<0.01	0.002

**Table 3:** Comparison of VAS scores.

Groups	*n*	5 min after analgesia	10 min after analgesia	30 min after analgesia
Analgesic group	45	3.42 ± 1.25	2.68 ± 0.87	1.41 ± 0.67
Non-analgesic group	45	8.19 ± 1.38	8.42 ± 1.17	8.28 ± 1.22
*t*-value	—	17.185	26.409	33.11
*P* value	—	<0.001	<0.001	<0.001

**Table 4:** Comparison of delivery mode and indomethacin use.

Groups	*n*	Vaginal assisted delivery	Vaginal normal delivery	Cesarean delivery	Use of indomethacin
Analgesic group	45	3.42 ± 1.25	2.68 ± 0.87	1.41 ± 0.67	23 (51%)
Nonanalgesic group	45	8.19 ± 1.38	8.42 ± 1.17	8.28 ± 1.22	12 (27%)
*t*-value	—	17.185	26.409	33.11	5.657
*P* value	—	<0.001	<0.001	<0.001	0.017

## Data Availability

No data were used to support this study.
